The article "Practical Research on Artificial Intelligence Algorithms, Paleontology, Data Mining, and Digital Restoration of Public Information" was retracted in 2023. Reasons: unreliable results or conclusions; concerns about the data; concerns about the results or conclusions; concerns about the peer review.

# Practical Research on Artificial Intelligence Algorithms, Paleontology, Data Mining, and Digital Restoration of Public Information

**DOI:** 10.1155/2022/3068686

**Published:** 2022-09-28

**Authors:** Guo Yan, Hong Xin

**Affiliations:** Digital Protection and Application of Paleontology Lab, Media and Animation College, Lu Xun Academy of Fine Arts, Dalian, China

## Abstract

This paper discusses the method of fossil digitization combining paleontology and art by using data mining. The aim of the study is to increase the creativity and vitality of museum exhibits and promote scientific exchange. The purpose of the study is to discuss how the interdisciplinary approach will benefit the communication of science and to realize the cooperative development of creative science popularization, art science popularization, dialogue science popularization, and communication science popularization through the cooperation between museums and institutions disseminating and researching science. The research method takes the Jehol Biota in western Liaoning Province of China as an example to explore the methods and approaches to transform museum resources into creative products. Through artificial intelligence data mining and digital reconstruction, data can be used for archaeological research but also for scientific popularization and scientific dissemination of the resources of art transformation. Research results: as the cornerstone to consolidate the digital development of society and economy, “the new infrastructure of artificial intelligence” will start a comprehensive digital transformation. Through the integration of multiple fields and disciplines, museums will change from resource dependence to focus more on market creation, which will promote museum's industry development.

## 1. Introduction

With the rapid development of information technology and the Internet, massive amounts of data have been generated explosively. Data mining refers to the process of searching for information hidden in a large amount of data through algorithms. How to effectively process and store these massive data and mine the hidden knowledge from these data is an important and meaningful work. In a broad sense, data mining is a kind of deep-seated data analysis method, which fuses artificial intelligence, data bases, machine learning, and statistics, to meet the demand for directional selection of a large amount of data. There are mainly ten methods in data mining, and we choose K-means and Naive Bayes as the main methods.

During the 23rd collective learning of the Central Political Bureau, General Secretary Jinping Xi commented, “There are cultural relics in museums, heritage on the vast land, and written words in ancient books. Let's make them alive” [1]. This paper uses the Jehol Biota of western Liaoning, China, as the main case study. We digitally restore the fossils and use front-projected holographic display technology and somatosensory interaction technology to construct sci-com *x* art exhibitions, which will be displayed in the science museum, cultural art museum, and outside of museums such as public places [2]. It is especially meaningful to the cultural protection and development in relatively less developed regions, which will open a new development path. From this, we integrate these ideas with science and technology, driving the research and development of this subject. We conduct inspiring, pioneering, and constructive research explorations.

Dr Carney utilized radiography and scanned the fossil of a well-preserved Archaeopteryx, which resulted in a series of images that display the internal structure of the specimen. The bones of Archaeopteryx were separated from surrounding rocks with computer modelling technique. The segmented bone data were built into 3D models and subsequently a mounted skeleton of Archaeopteryx. Lastly, the locomotion of Archaeopteryx was simulated using an animation technique with reference to research on reptile kinematics. This research has provided a framework on the methodology and techniques used in the reconstruction of fossil animals, which has a high application and research value.

In China, integration of science and art has been implemented in practice, maximizing the influence of science education from an aesthetic and artistic perspective. For example, the Shanghai Science and Technology Museum, in collaboration with several museums and institutes, has hosted a science cultural exhibition of “The Belt and Road Initiative,” called ‘The students surpass the teacher—the origin, development and exchange of blue and white porcelain'. This exhibition did not only showcase the development, culture, and art appreciation of blue and white pottery but also its production and related scientific development, showing integration of science and art to the public. In addition, Dr Yan Liang at the University of Science and Technology of China has shot a video series called “Beautiful Chemistry,” explaining the beauty of science from the art perspective, aiming to get more children interested in chemistry. Some artists have collaborated with scientists and musicians to transform meteorological data into a music score. The music score was performed in a concert, hoping to call on people to pay attention to climate change by artistically visualizing the data [3]. Under the influence of national policies, paleontology, and knowledge of fossils, it can be understood by more people in a dynamic and diverse way. It is not only a good way to express propaganda but a pregnant chance to develop the integrated disciplines and improve more students' comprehensive learning ability. Besides, through a more digital design, we can break the time limit and improve the learning efficiency by a panoramic experience.

## 2. Digital Protection of the Jehol Biota of Western Liaoning

### 2.1. Current Status of Protection and Limitations

Currently, the protection of western Liaoning fossils is mainly dominated by the traditional method, which is the storage of specimens in a temperature-controlled and humidity-controlled environment. Following excavation, the fossils are graded by the national authority; fossil localities are designated as nature reserves for overall protection. Specimens are valuable to scientific research, but relevant cultural industry development is absent. The Chaoyang National Geopark, for example, protects the fossil excavation site by building a pavilion in situ, using it for sightseeing. Due to the increased number of visitors and influence by natural conditions, the inner wall of the fossil layers has started to peel off to a greater extent as time goes by. In terms of product development, the products sold in the museum store have no brand awareness, which suppresses a consumer's desire to buy. The most popular products of fossils are fish and insects, but such resources are limited, so a creative transformation is necessary for sustained development.

On the other hand, apart from exquisitely preserved animal and plant fossils, there are abundant fragmentary fossils, animals in particular. These scarce fossils are also part of the important scientific information but are usually overlooked. Farmers at the Sihetun of Beipiao, western Liaoning (the locality of Sinosauropteryx) are known to have used fossils in wall construction. Thus, scientific communication and promotion are also of paramount importance in fossil protection.

### 2.2. Protection Methods and Procedures

This project uses one of the technologies of artificial intelligence (AI), data mining, to enrich the background information and build 3D models, which effectively improve the accuracy of modelling.

Digital protection of the Jehol Biota of western Liaoning could be implemented in two aspects, namely collection and classification. 3D models are constructed with reference to raw research data and compiled into a 3D model database of western Liaoning Jehol Biota. The restored 3D models are valuable to both product development and research. We use the specimen of Nurhachius luei as an example to demonstrate our proposed methods and procedures. Firstly, we created a line drawing based on the specimen (Figure 1). Secondly, we generated a restored 3D model (Figure 2). This fossil is a holotype specimen with clearly visible bones, such that data extraction and restoration are relatively direct. However, for relatively fragmentary specimens, comparisons with closely related taxa in the database are needed to aid restoration. With the development of AR (augmented reality) and VR (virtual reality), more discipline and knowledge will be transmitted by 3D, and 3D has become one of the most prevalent technologies today without a doubt. By using 3D models, the project can give people a more intuitive and three-dimensional experience.

## 3. Data Mining Classification Algorithms

### 3.1. Support Vector Machines

A support vector machine is a supervised two-class classification model. The classification process is actually to find the optimal classification surface. It has been originally applied to the linearly separable case, and it has now been extended to the nonlinear case with strong generalization capabilities [5, 6].

The linear classifier is the original form of SVM [7]. It is assumed that the value corresponding to the upper point is *y* = 1, and the value corresponding to the lower point is *y* = −1. The classification surface is expressed as *f*(*x*)=*u*^*o*^*x*+*t*. If *f* (*x*) is less than 0, it is judged that *x* is for the lower point, if *f* (*x*) is greater than 0, it is judged that *x* is above, and if *f* (*x*) is equal to 0, it is judged that *x* is on the classification plane.

Figure 3 shows two classification straight lines. The larger the gap, the more accurate the classification [8]. If the gap distance is K, then

(1) $$\begin{array}{c} K=\frac{2}{\sqrt{u•u}}=\frac{2}{\left\|u\right\|}\text{.} \end{array}$$

The point on the edge of the line is the support vector, then the expression of the support vector is as follows: [9, 10]

(2) $$\begin{array}{c} yf\left(x\right)=y\left(u^{o}x+t\right)=1\text{.} \end{array}$$

After obtaining the support vector, the classification problem is transformed into finding the maximum N: [11, 12]

(3) $$\begin{array}{c} \max\frac{1}{\left\|u\right\|}\Leftrightarrow \frac{{\left\|u\right\|}^{2}}{2}\text{.} \end{array}$$

According to *y*_*a*_(*x*)(*u*^*o*^*x*+*t*) ≥ 1, *a*=1,2,…, *m* under the constraint condition, formula (3) is transformed into

(4) $$\begin{array}{c} \frac{{\left\|u\right\|}^{2}}{2},s.t.y_{a}\left(u^{o}x_{a}+t\right)\geq 1,a=1,2,\ldots ,m\text{,} \end{array}$$

transform into

(5) $$\begin{array}{c} L\left(u,t,\varpi \right)=\frac{{\left\|u\right\|}^{2}}{2}-\overset{m}{\underset{a=1}{\sum }}\varpi_{a}\left(y_{a}\left(u^{o}x_{a}+t\right)-1\right)\text{.} \end{array}$$

Converted to the problem of optimizing bivariate by Lagrangian binary and differentiating u: [13, 14]

(6) $$\begin{array}{c} \frac{\partial L}{\partial t}=0\Rightarrow u-\overset{m}{\underset{a=1}{\sum }}\varpi_{a}y_{a}x_{a}=0\text{.} \end{array}$$

Redifferentiate

(7) $$\begin{array}{c} \frac{\partial L}{\partial t}=0\Rightarrow \overset{m}{\underset{a=1}{\sum }}\varpi_{a}y_{a}=0\text{.} \end{array}$$

Substituting equations (6) and (7) into equation (5), the dual variable expression can be obtained as follows:

(8) $$\begin{array}{c} L\left(u,t,\varpi \right)=\overset{m}{\underset{a=1}{\sum }}\varpi_{a}-\frac{1}{2}\overset{m}{\underset{a,b=1}{\sum }}\varpi_{a}\varpi_{b}y_{a}y_{b}x_{a}^{o}x_{b}\text{.} \end{array}$$

The final question turns into

(9) $$\begin{array}{c} \begin{array}{c} \max_{\varpi }\overset{m}{\underset{a=1}{\sum }}\varpi_{a}-\frac{1}{2}\overset{m}{\underset{a,b=1}{\sum }}\varpi_{a}\varpi_{b}y_{a}y_{b}x_{a}^{o}x_{b},\\ s.t.\varpi_{a}\geq 0,a=1,2,\ldots ,m,\overset{m}{\underset{a=1}{\sum }}\varpi_{a}y_{a}=0. \end{array}\text{.} \end{array}$$

In the case of linear inseparability, there are usually two solutions: one is to use curve classification, and the other is to use straight lines, but the premise is that the misclassified points can be accommodated [15–17].

A penalty function is set for each outlier point, which is expressed as the distance from the outlier point to the correct classification boundary [18, 19]. Then, in the case of linear separability, the penalty function and constraints can be added, which can be expressed as

(10) $$\begin{array}{c} \frac{{\left\|u\right\|}^{2}}{2}+S\overset{M}{\underset{a=1}{\sum }}\mu_{a},s.t.\varpi_{a}\text{(}y_{a}\left(u^{o}x_{a}+t\right)\geq 1-\mu_{a},\mu_{a}\geq 0\text{.} \end{array}$$

*D*∑*a*=1*Mμ*_*a*_ is the penalty function, *M* is the total number of data points, S is the weighting coefficient, and the larger the S, the more correct the classification result.

Transform (10) using Lagrangian duality as follows:

(11) $$\begin{array}{c} \begin{array}{c} \max_{\varpi }\overset{m}{\underset{a=1}{\sum }}\varpi_{a}-\frac{1}{2}\overset{m}{\underset{a,b=1}{\sum }}\varpi_{a}\varpi_{b}y_{a}y_{b}x_{a}^{o}x_{b},\\ s.t.0\leq \varpi_{a}\leq S,a=1,2,\ldots ,m,\overset{m}{\underset{a=1}{\sum }}\varpi_{a}y_{a}=0. \end{array}\text{.} \end{array}$$

For the linearly inseparable case, the classification function is set as

(12) $$\begin{array}{c} f\left(x\right)=\overset{m}{\underset{a=1}{\sum }}u_{a}\theta_{a}\left(x\right)+t\text{.} \end{array}$$

Through dual transformation, it can be transformed into

(13) $$\begin{array}{c} f\left(x\right)=\overset{m}{\underset{a=1}{\sum }}\varpi_{a}y_{a}\langle \theta \left(x_{a}\right),\theta \left(x\right)\rangle +t\text{.} \end{array}$$

〈*θ*(*x*_*a*_), *θ*(*x*)〉 can be replaced by an appropriate kernel function without increasing the number of callable parameters to solve the optimal problem:

(14) $$\begin{array}{c} \begin{array}{c} \max_{\varpi }\overset{m}{\underset{a=1}{\sum }}\varpi_{a}-\frac{1}{2}\overset{m}{\underset{a,b=1}{\sum }}\varpi_{a}\varpi_{b}y_{a}y_{b}\langle \theta \left(x_{a}\right),\theta \left(x_{b}\right)\rangle ,\\ s.t.\varpi_{a}\geq 0,a=1,2,\ldots ,m,\overset{m}{\underset{a=1}{\sum }}\varpi_{a}y_{a}=0. \end{array}\text{.} \end{array}$$

The high-dimensional space corresponding to the low-dimensional space grows exponentially. To reduce the computational difficulty, the kernel function *Q*(*x*_*a*_, *x*_*b*_) needs to be introduced.

Assuming that there are two vectors *x*_1_=(*ς*_*a*_, *ς*_*b*_)^*o*^ and *x*_2_=(*ς*_*a*_, *ς*_*b*_)^*o*^ in the two-dimensional space, the expression after matching to the five-dimensional space through the matching function *θ* (*x*) is

(15) $$\begin{array}{c} \langle \theta \left(x_{1}\right),\theta \left(x_{2}\right)\rangle =\varsigma_{1}\gamma_{1}+\varsigma_{1}^{2}\gamma_{1}^{2}+\varsigma_{2}\gamma_{2}+\varsigma_{2}^{2}\gamma_{2}^{2}+\varsigma_{1}\varsigma_{2}\gamma_{1}\gamma_{2}\text{.} \end{array}$$

If you directly consider

(16) $$\begin{array}{c} {\left(\langle x_{1},x_{2}\rangle +1\right)}^{2}=2\varsigma_{1}\gamma_{1}+\varsigma_{1}^{2}\gamma_{1}^{2}+2\varsigma_{2}\gamma_{2}+\varsigma_{2}^{2}\gamma_{2}^{2}+2\varsigma_{1}\varsigma_{2}\gamma_{1}\gamma_{2}+1\text{.} \end{array}$$

Equations (15) and (16) are only different in the linear scale of dimensions and have a constant dimension. In fact, the following calculations are performed first:

(17) $$\begin{array}{c} \theta \left(X_{1},X_{2}\right)={\left(\sqrt{2}X_{1},X_{1}^{2},\sqrt{2}X_{2},X_{2}^{2},\sqrt{2}X_{1}X_{1}^{2},1\right)}^{Q}\text{.} \end{array}$$

The result is consistent with 〈*θ*(*x*_1_), *θ*(*x*_2_)〉. Therefore, mapping from two-dimensional space to five-dimensional space and then calculating the inner product is consistent with calculating directly in two-dimensional space and then reflecting the result to five-dimensional space. In the second calculation process, the inner product function of equation (16) is the kernel function, which is given as follows:

(18) $$\begin{array}{c} Q\left(x_{1},x_{2}\right)={\left(\langle x_{1},x_{2}\rangle +1\right)}^{2}\text{.} \end{array}$$

Then, the classification function of formula equation (13) should be expressed as

(19) $$\begin{array}{c} f\left(x\right)=\overset{m}{\underset{a=1}{\sum }}\varpi_{a}y_{a}Q\left(x_{a},x\right)+t\text{.} \end{array}$$

The extremum optimization problem of equation (14) is expressed as

(20) $$\begin{array}{c} \begin{array}{c} \max_{\varpi }\overset{m}{\underset{a=1}{\sum }}\varpi_{a}-\frac{1}{2}\overset{m}{\underset{a,b=1}{\sum }}\varpi_{a}\varpi_{b}y_{a}y_{b}Q\left(x_{a},x_{b}\right),\\ s.t.\varpi_{a}\geq 0,a=1,2,\ldots ,m,\overset{m}{\underset{a=1}{\sum }}\varpi_{a}y_{a}=0 \end{array}\text{.} \end{array}$$

## 4. Application of the Digital Data of the Jehol Biota of Western Liaoning

### 4.1. Current Status of the Application and Existing Problems

Iconic palaeotological museums in China such as the Paleozoological Museum of China and the Nanjing Museum of Paleontology mostly focus on the display of existing resources, supplemented by popular science talks to promote knowledge and information related to paleontology. Digital art is widely applied in various fields, including the exhibitions of numerous museums around the globe [16]. Paleontological museums are also exploring this way of transformation. It is important to maintain its characteristics while integrating with other disciplines, as well as transforming museum resources to more creative-based while protecting the heritage. These are the problems that need to be considered.

### 4.2. Application Methods and Procedures

The equations are an exception to the prescribed specifications of this template. You will need to determine whether or not your equation should be typed using either the Times New Roman or the Symbol font (please no other font). To create multileveled equations, it may be necessary to treat the equation as a graphic and insert it into the text after your paper is styled.

This paper uses an application-oriented approach throughout this study, including data collection. Based on facts and combined with artistic techniques, we produce basic models that could be utilized in future exhibitions. The final output will be presented in the forms of online popular science education and offline popular science experience.

For example, the fossil of Nurhachius luei was collected, three-dimensionally restored, modelled, and rendered (Figure 4). This could be used for flow experience with 4 K rendering. Muscle reconstruction is also an important component in scientific research and knowledge in future exhibitions integrating science and art (Figure 5). The protection of western Liaoning fossils wants to illustrate the bone structure of palaeobios and their muscles and feathers, and the demand of propagandizing scientific knowledge can be satisfied effectively. The muscle reconstruction can be detailed in the illustration of palaeobios.

Online popular science education: mobile APPs facilitate the continuous transmission of scientific knowledge, combining texts, images, animations, games, and relevant output. They could deliver messages to users via multiple forms in an interesting, creative, interactive, multidimensional, and high-efficiency way (Figure 6). The usage data could be used to build a database that reflects user needs, which helps us improve online and offline services. Online teaching has become mainstream under the influence of COVID-19, although without epidemic, online interaction has become more and more prevalent with the help of Internet and computer technology. Online teaching is not only good for epidemic prevention and control, but they also give a chance to show the comprehensive technology.

Offline popular science experience: it is an innovative mode of exhibition, allowing the exhibits to “walk” out of the museum. “The walking prehistoric animals” is a collaborative science-art project by the Lu Xun Academy of Fine Arts and Chaoyang City Government of western Liaoning. It is an exploration of integrating paleontological popular science and art. The exhibits are all in digital image format, which are easy to build and dismantle. There will be more exhibits using other technologies in the future experience hall, such as AR, VR, and Hologram, as well as numerous products that meet the various needs of the consumers. Visitors will travel through time and space and walk with dinosaurs (Figure 7). They will learn and play while enjoying the exhibition.

## 5. Conclusions

With the rapid development of computer science and technology, the channels of data generation are more extensive, and how to effectively store and utilize the vast ocean of data is an important task. “New Infrastructure,” as a cornerstone for consolidating the digital development of the socio-economy, will open up a comprehensive digital transformation. Through multifield and multidisciplinary integration, museums will change from being resource-dependent to focusing more on market creation, which will promote the development of this industry. With the development of the Internet and technology, online and offline environments will connect with “no delay.” The current interaction is between a human and the digital models of fossils, while the one in the future will be between a human and a virtual environment. The character in the virtual environment will be controlled by another user. The user can enrich the information of the “character,” which allows them to send out information while compiling them. They will become a participant in the virtual world but not only a recipient of science knowledge. The resources belong to the public; everyone is also a provider of knowledge. Digital paleontological reconstruction from a cultural industry perspective is an exploration that will benefit popular science education. In this case, we have found and made a further exploration to drive public attention on comprehensive digital exhibition. The digital design methods have provided a new way to protect fossils or other ancient resources. The public is the producer of cultural products and cultural creativity. Their demand is an important basis for the update and iteration of the cultural industry. Public welfare is one of the attributes of culture. Using modern technologies, the transmission scope is enlarged. Since the efficiency of resource sharing is raised, the cost of science communication is lowered, maximizing the value of the exhibition. All in all, this will achieve the ultimate aim of paleontological resource protection, as well as driving regional cultural and economic development.

## Figures and Tables

**Figure 1:** Specimen of Nurhachius luei (adapted from Zhou et al.) [4].

**Figure 2:** 3D restoration of Nurhachius luei.

**Figure 3:** Two classification cases.

**Figure 4:** Rendered model of the restored skull of Nurhachius luei.

**Figure 5:** Muscle reconstruction of Nurhachius luei.

**Figure 6:** A scene in the popular science game “Fly to the sky.”

**Figure 7:** Ecological reconstruction of Jehol Biota by rendering of 3D models.

## Data Availability

The data used to support the findings of this study are available from the corresponding author upon request.

## References

[1] Xiansong N. (2017). Cross border integration of science and art. *Development Herald*.

[2] Xuxing J., Xiaolin W. (2001). The origin of feathered dinosaurs and birds. *Journal of the Chinese Academy of Sciences*.

[3] Luo X. (2020). Discussion on the basic process of digitization and Representation of cultural relics— based on the digitization work of the cultural relics of Liangzhu museum. *Study on natural and cultural heritage*.

[4] Zhou X., Pêgas R. V., Leal M. EC., Bonde N. (2019). Nurhachius luei, a new istiodactylid pterosaur (Pterosauria, Pterodactyloidea) from the Early Cretaceous Jiufotang formation of Chaoyang City, Liaoning province (China) and comments on the Istiodactylidae. *PeerJ*.

[5] Jianqing Z. (2017). Reflection on the restoration of Chinese dragon and bird. *Operation and management*.

[6] Buczak A. L., Guven E. (2016). A Survey of data mining and machine learning methods for Cyber Security Intrusion Detection. *IEEE Communications Surveys & Tutorials*.

[7] Xu L., Jiang C., Wang J., Yuan J., Ren Y. (2014). Information Security in Big data: Privacy and data mining. *IEEE Access*.

[8] Kavakiotis I., Tsave O., Salifoglou A., Maglaveras N., Chouvarda I. (2017). Machine learning and data mining methods in Diabetes research. *Computational and Structural Biotechnology Journal*.

[9] Chaurasia V., Pal S. (2017). A Novel approach for Breast Cancer Detection using data mining techniques. *Social Science Electronic Publishing*.

[10] Chen W., Panahi M., Pourghasemi H. R. (2017). Performance evaluation of GIS-based new ensemble data mining techniques of adaptive neuro-fuzzy inference system (ANFIS) with genetic algorithm (GA), differential evolution (DE), and particle swarm optimization (PSO) for landslide spatial modelling. *Catena*.

[11] Yan X. S., Zheng L. (2017). Fundamental analysis and the Cross-Section of Stock Returns: a data-mining approach. *Review of Financial Studies*.

[12] Emoto T., Yamashita T., Kobayashi T. (2017). Characterization of gut microbiota profiles in coronary artery disease patients using data mining analysis of terminal restriction fragment length polymorphism: gut microbiota could be a diagnostic marker of coronary artery disease. *Heart and Vessels*.

[13] Hong H., Tsangaratos P., Ilia I., Liu J., Zhu A. X., Chen W. (2018). Application of fuzzy weight of evidence and data mining techniques in construction of flood susceptibility map of Poyang County, China. *Science of The Total Environment*.

[14] Wu W., Peng M. (2017). A data mining approach combining $K$ -means Clustering with Bagging Neural Network for Short-Term Wind Power Forecasting. *IEEE Internet of Things Journal*.

[15] Zheng L., Hu W., Min Y. (2015). Raw Wind data Preprocessing: a data-mining approach. *IEEE Transactions on Sustainable Energy*.

[16] Marozzo F., Talia D., Trunfio P. (2018). A Workflow Management system for scalable data mining on Clouds. *IEEE Transactions on Services Computing*.

[17] Rupesh W., Sagar J., Rahul S. (2017). An internal Intrusion Detection and protection system by using data mining and Forensic techniques. *IEEE Systems Journal*.

[18] Karimi M. B., Isazadeh A., Rahmani A. M. (2017). QoS-aware service composition in cloud computing using data mining techniques and genetic algorithm. *The Journal of Supercomputing*.

[19] Moustakas A. (2017). Spatio-temporal data mining in ecological and veterinary epidemiology. *Stochastic Environmental Research and Risk Assessment*.

[20] Sacks R., Wang Z., Ouyang B., Utkucu D., Chen S. (2022). Toward artificially intelligent cloud-based building information modelling for collaborative multidisciplinary design. *Advanced Engineering Informatics*.

[21] Manimuthu A., Venkatesh V. G., Raja Sreedharan V., Mani V. (2022). Modelling and analysis of artificial intelligence for commercial vehicle assembly process in VUCA world: a case study. *International Journal of Production Research*.

[22] Thon C., Böttcher A. C., Möhlen F., Yu M., Kwade A., Schilde C. (2022). Multi-modal framework to model wet milling through numerical simulations and artificial intelligence (part 1). *Chemical Engineering Journal*.

[23] Li H., Li X., Yuan F. (2022). Knowledge-driven based three-dimensional prospectivity modeling of Fe–Cu skarn deposits; a case study of the Fanchang volcanic basin, anhui province, Eastern China. *Ore Geology Reviews*.

